This article has been retracted.

# Wireless Sensor Technology-Based Physical Education Teaching Evaluation

**DOI:** 10.1155/2022/3544457

**Published:** 2022-07-07

**Authors:** Wei Feng

**Affiliations:** Sanquan College of Xinxiang Medical University, Henan 453000, China

## Abstract

A wireless sensor network (WSN) is a group of geographically scattered and specialized sensors to monitor and record variables related to environmental and storing the obtained data in a vital location. These networks have applications and can be utilized in different research domains including physical education where error prediction is assumed as one of the core issues. Thus, careful attention is required from the researcher to provide reliable and accurate prediction models. Thus, aiming the shortage of large prediction error in the physical education evaluation, which is based on the BP neural network and wireless sensor technology, a combination of AFP and questionnaire survey method is proposed in order to improve the accuracy and predictability of evaluation, according to the characteristics of different evaluation subjects. We select the evaluation index system as the input of wireless sensor technology and then use the principle of genetic algorithm to select the optimal individual and optimize the initial parameters of wireless sensor technology to establish the evaluation model of physical education quality. Through the training and testing of sample data, it is shown that the model greatly improves the accuracy of physical education quality evaluation and has a good application prospect in physical education evaluation.

## 1. Introduction

A wireless sensor network is an internet-connected system of linked devices that can be accessed from anywhere in the world. The main goal of WSNs is to make people's lives more complex, versatile, and accessible to a wide range of devices all around the world. This paradigm has a wide range of applications, including intelligent transportation and logistics, health care, smart environments (home, workplace, and plants), and personal and social domains. WSN devices may interact not just with one other within range, but also with external devices via a gateway device to send and receive data. This network has a vast application domains ranging from ordinary medical or health sector to physical education. In these networks, a base station or sink seems to be a connection point between users and the network. By inserting some requests and retrieving results from the sink, it can transform some essential information from the network. A wireless sensor network often has tens of thousands of sensor nodes which are capable of collecting various kinds of information. These sensors can work as neurons which are the basic unit of the neural network that is used in various projects for the evaluation of the quality in the physical education.

Physical education quality evaluation is a systematic project with heavy workload and cumbersome statistics. Based on the powerful nonlinear data processing ability of the neural network, it is mainly used as the main algorithm for teaching quality evaluation. In view of these shortcomings, domestic scholars have proposed AFP algorithm, direct value method, learning vector quantization algorithm, particle swarm optimization algorithm, principal component analysis method, multilayer wireless sensor technology algorithm, support vector machine algorithm, quantum neural network algorithm, etc. The combination of algorithms effectively improves the reliability and accuracy of physical education quality evaluation. These improvement methods are mainly divided into the following two types: ① using the AFP or principal component analysis method to screen out those that have an important impact on the evaluation results, it is used as the input of wireless sensor technology to improve the noncorrelation of the input independent variables of wireless sensor technology; ② use learning vector quantization, particle swarm optimization and support vector machine, and other algorithms to improve structure of the network or error model of wireless sensor technology to increase speed and accuracy of the convergence and prediction, respectively. A commonly used model of the neural network is the back propagation (BP) neural network algorithm, which is based on the idea of multiple layer structure and is educated in fashion to effectively make use of the error back propagation algorithm. This algorithm has the capacity to resolve numerous possible issues, like the one carried out in this paper, if it is combined maturely with another algorithm.

In this paper, according to the characteristics of the teaching authorities, teaching supervisors, teaching peers, and students in teaching evaluation, the AFP (AHP) and the questionnaire survey method are comprehensively used to screen important evaluation indicators as a multilayer feedforward (back propagation, BP) neural network input. In next phase, we use genetic algorithms (GAs) to optimize the initial weights and thresholds of BP neural network and improve the accuracy of physical education quality evaluation through the improved BP neural network model. This model is assumed to be efficient in terms of accuracy and precision ratio.

The rest of the paper is organized as given in the following.

Evaluation of wireless sensor technology is reported in the next section where it is clearly defined how these technologies are vital in resolving various issues related to the problem domain. More importantly, weight index calculation of this technology is reported as well. In Section 3, an improved version of the traditional BP neural network, which is already available and is primarily based on the idea or algorithm of the genetic algorithm, is reported. Results of the proposed neural network model and discussions are provided in Sections 4 and 5, respectively. Lastly, conclusion is given.

## 2. Evaluation of Wireless Sensor Technology

The analytic hierarchy process (AHP) is used to calculate the importance weights of the evaluation indicators and screen the important evaluation indicators [1] in order to address the characteristics of wireless sensor technology sports teaching evaluation that the teaching department and supervision experts are familiar with the teaching rules and grasp the evaluation importance level is accurate. A wireless sensor communicates with other nodes via the communication unit, which includes a transceiver that serves as both a transmitter and a receiver. Radio frequency, optical (laser), or infrared transmission media are all possibilities for wireless communication. Finally, the two types of data are integrated to screen critical signs for use as input in the next BP neural network assessment model [2].

### 2.1. Wireless Sensor Technology Calculation Index Weight

First, establish a hierarchical structure model according to the target layer, the criterion layer (6 first-level indicators), and the subcriteria layer (24 second-level indicators) based on the initially established wireless sensor technology evaluation index content system. The indicators of the criterion layer are compared pairwise [3]. In this paper, the teaching authorities and supervising experts who are familiar with the quality evaluation of physical education are used to determine the score, and a judgment matrix A is constructed. Evaluation of quality is a controlled process where a third party, generally an administrator or a member of the QM/QA team, evaluates interaction of an agent that is based on key criteria stated in a quality form. In comparison to the 9-quantile scaling methodology and the 1.354 scaling method, the golden section 0.618 is used as the AFP to assess the disadvantages of distortion, and the assignment criteria for the components in the judgment matrix are listed in Table 1;

Then, using Matlab software programming, the eigenvectors corresponding to the maximum eigenvalues *λ*max and *λ*max of each judgment matrix are obtained, respectively [4], and the consistency check is completed, and the maximum eigenvector obtained by normalization is the weight of each required evaluation index.; finally, calculate the relative importance of the same level to the total evaluation results of teaching quality [5, 6], conduct consistency test on the judgment matrix from high to low, get the comprehensive weight of each index, and finally screen out 12 evaluation indicators with higher weights, section 0.618.

### 2.2. Questionnaire Survey Statistics Concern Indicators

Surveys of questionnaire require to be utilized or follow a set of question, which is preferably in a sequential order, to fetch statistical data about a population's individualities, beliefs, characteristics, and behaviors. In order to investigate and count the attention of teaching peers and students to the evaluation index items [7], the preliminarily established evaluation index content system was made into a questionnaire, and it was required to select 12 most concerned evaluation points from the 24 secondary indicators. Finally, 114 valid questionnaires from teaching peers and 397 valid responses from students were collected, and the 12 indicators with the highest attention were obtained from statistics.

### 2.3. Important Indicators of Wireless Sensor Technology Screening

The AHP calculates the weight of the indicators and the attention of the indicators in the questionnaire survey and compares the 12 indicators calculated by these two methods. There are 8 identical and 4 different. It can be seen that the important indicators selected from different angles basically overlap [8], but there are also a small number of indicators that are different due to different evaluators' cognitive laws and reference angles. In this paper, the results of the two methods are combined, and the same 8 indicators are used as the input of the next neural network evaluation model. The specific evaluation indicators are shown in Table 2.

## 3. GA-Enabled BP Neural Network

This paper uses the principle of genetic algorithm GA to select the optimal individual, selects the optimal initial weights and thresholds for the wireless sensor technology network, and constructs an improved wireless sensor technology network to improve the prediction accuracy of the wireless sensor technology network evaluation model [9]. A genetic algorithm is a search heuristic-enabled approach based on natural hypothesis of selection presented by Charles Darwin, or a natural selection inspired metaheuristic, which is considered as a portion or subpart of algorithms known as evolutionary particularly in the domain of computer science. It is important to note that it is exhibited after the scheme, i.e., natural selection, where it is evident that most optimal, i.e., fittest, parts or agents or individuals are chosen to represent a reproduction in such a way that it can produce individuals of next generation [10].

### 3.1. Steps to Construct an Improved Wireless Sensor Technology Network

The steps of improving wireless sensor technology network based on GA are shown in Figure 1.

① Determine the wireless sensor technology network structure. Determine the topological structure of the wireless sensor technology network, including number of input and output nodes and number of network and hidden layers, respectively.
② Calculate the number of network weights and thresholds, that is, the length. Assuming that the network determined in step ① is a 3-layer structure of *x*-*y*-1, the calculated network weights are (*x∗y* + *y*), the network threshold is (*y* + 1), and the total number or length is shown in the following formula:
  (1) $$\begin{array}{c} \text{LEN}=\left(x*y+y\right)+\left(y+1\right). \end{array}$$
③ Population initialization of the genetic algorithm: determine the length of individual code as LEN, choose the binary method or the real number method for individual code, and determine the operating parameters such as population size, probability of crossover, and mutation.
④ Take the error sum of wireless sensor technology network training as the fitness function. Dataset reserved for training must be utilized for the training of network [11], and take the error's absolute value between output (actual) and expected output as separate value of fitness *F*, and the calculation is shown in the following formula:
  (2) $$\begin{array}{c} F=k\sum_{i=1}^{n}\left(y_{i}-o_{i}\right), \end{array}$$
where *n* represents output nodes or devices in networks; *y*_*i*_ parameter is used to represent wireless technology's *i*^th^ node's expected output value; *o*_*i*_ is the *i*^th^ node's predicted output; *k* is the coefficient.
⑤ Crossover, selection, and mutation operations of the genetic algorithm: the calculation formulas are formula (3), formula (4), and formula (5):
  (3) $$\begin{array}{c} \text{pselect}=\frac{f_{i}}{\sum_{j=1}^{N}f_{i}}. \end{array}$$
In the formula, pselect is the probability of the individual node selection; *f*_*i*_=(*k*/*F*_*i*_), *F*_*i*_ are the fitness values of single *i*, and smaller value will produce better *k* coefficient; population's individuals are reported by *N*:
  (4) $$\begin{array}{c} a_{mj}=a_{mj}\left(1-b\right)+a_{nj}b,\\ a_{nj}=a_{nj}\left(1-b\right)+a_{mj}b. \end{array}$$
The crossover operation technique of the *m*^th^ and *n*^th^ chromosomes at the *j* location utilising the real number coding method is represented by formula (4). *b* is a number between 0 and 1:
  (5) $$\begin{array}{c} a_{ij}=a_{ij}+\left(a_{ij}-a_{\max}\right)*f\left(ga\right),\text{rand}>0.5,\\ a_{ij}=a_{ij}+\left(a_{\min}-a_{ij}\right)*f\left(ga\right),\text{rand}<0.5. \end{array}$$
Equation (5) is a process to choose *j*^th^ gene *a*_*ij*_ of individual at position *i*^th^, and mutation operation is applied. *a*_*ij*_ gene is the upper bound of *a*_max_; *a*_*m*in_ is the lower bound of gene *a*_*ij*_; *f*(*ga*)=*r*(1 − (*ga*/*ga*)_index)^2^, where variable *r* represents random number; current iteration is *ga*; *ga* _index is the maximum evolution number; rand is a random number between [0,1].
⑥ Choose the most qualified person. The ideal individual is chosen based on the fitness value once the number of evolution iterations has been finished.
⑦ Determine the best weights and thresholds. The ideal individual's code is returned to the wireless sensor technology network's optimal beginning weight and threshold.
⑧ Improve the BP neural network's training and testing. Train the network with the training data, compute the mean square error MSE, and end training when the error is less than the goal value. Use the model for the next prediction application.

### 3.2. Analysis of the Network Effect of Improved Wireless Sensor Technology

We compared the traditional BP neural network and the improved wireless sensor technology network based on GA, and fitting binary nonlinear functions *Y*=*x*_1_^2^+*x*_2_^2^+*x*_1_*∗x*_2_, respectively, to understand the effect of the improved GABP neural network. According to the structure of the function, choose 2-5-1 3-layer BP neural network structure [12]. The application creates 2000 pairs of input and output data at random between [0, 5] using the Matlab platform, with the first 1900 groups serving as training samples and the final 100 serving as testing samples.  Figure 2 shows a comparison of the prediction error curves of the two networks. As can be seen, the optimised GABP prediction error has substantially improved, making it perfectly suitable for use in assessing physical education quality.

## 4. Training and Testing of Improved Wireless Sensor Technology Models

In the solving problems like this one in this paper, training and testing of the underlined model are very important and these processes should be carried out in such as fashion to ensure maximum chances of accuracy and precision. Moreover, appropriate measure must be taken into account while carrying out these steps.

### 4.1. Source of Sample Data

In order to test the performance of the improved wireless sensor evaluation model, a simulation experiment was carried out on the Matlab platform. The sample data come from the physical education evaluation scores of 85 teachers [13].

According to the 8 important indicators screened out above, students are organized to evaluate and score the physical education teaching of teachers. In practice, students often score relatively high and cannot grasp the size of the score. The internal consistency is better. In the way of the Kerte five-point scale, the students choose the options of “Very Satisfied,” “Satisfied,” “General,” “Dissatisfied,” and “Very Dissatisfied” for each indicator, and then the computer will automatically convert the corresponding score [14]. In addition, we calculate the average score as the final score of this indicator; in order to ensure the validity of the sample data and the prediction accuracy of the neural network, the scientific and accurate output expected value is very important [15]. Therefore, this paper adopts the comprehensive score of each teacher's multiple lectures by the teaching authority and supervision experts as the expected value output of the wireless sensor technology network; finally, the original data need to be normalized.

### 4.2. Implementation of the Improved Wireless Sensor Technology Model

The number of input nodes of the wireless sensor technology network is decided to be 8 based on the main indicators screened above, and the complete score is utilized as the final assessment result for the evaluation of physical education quality. As a result, there is just one output node. Refer to [16] if a three-layer network configuration is used. Use the trial-and-error process to figure out that there are ten hidden layer nodes. The first 50 groups of data in the sample are utilized for network training, while the final 25 groups of data are used for output prediction.

The key code to realize the prediction of the improved wireless sensor evaluation model in Matlab is as follows:

  net = newff (a __trainn, *t* __trainn, [ 10,1], { 'tansig', pxuirelin'}, 'trainlm'); % Establish a wireless sensor technology network and use the LM algorithm to optimize the back propagation error model.
  ga_index = 20; % Genetic algorithm evolution algebra is the number of iterations.
  size _index = 10; % genetic algorithm population size is 10.
  pcross = [0.3]; % genetic algorithm crossover probability is 0.3.
  pmutation = [0.2]; % genetic algorithm mutation probability is 0.2.
  Individuals (I) = select (individuals, size _index); % genetic algorithm selection operation.
  Ichrom = cross (lengthchrom, pcross, I.chrom, size_index, range); % genetic algorithm cross operation.
  Ichrom = mutation(lengthchrom,pmutation, I.chrom, size _jindex, *i*,ga_index, range); % genetic algorithm mutation operation.
  NET.iw{ 1,1 } = reshape (q1, hidenum, inputnum); % assign the weight amid the optimal hidden & input layers in network.
  NET.lw 2,1 } = reshape (q2, outputnum, hidenum); % assign the weight amid the optimal hidden & input layers in network.
  NET.b{ 1 } = reshape (f1, hidenum, 1); % assign the optimal threshold amid the optimal hidden & input layers in network.
  NET.bi2} = *f*2; % Assign the threshold amid the optimal hidden & input layers in network.
  NET.trainparam.lr = 0.1; % network learning rate 0.1.
  NET.trainparam.epochs = 200; % network iterations 200 times NET.trainparam.goal = le-5; % network learning goal 1e-5.
  NET = train(NET, a_trainn, t_trainn); % train BP neural network t_testn = sim(net, a_testn); % test BP neural network.

### 4.3. Results Comparison and Analysis

The wireless sensor evaluation model without screening important evaluation indicators, the single-hidden-layer wireless sensor evaluation model with screening indicators, and the dual-hidden-layer wireless sensor screening indicators are chosen to evaluate the physical education quality evaluation model based on the wireless sensor technology physical education evaluation research.  Figure 3 depicts the prediction errors of multiple sensor assessment models after they have been compared and evaluated.

By comparing and analyzing the simulation results, the following conclusions can be drawn:

① Wireless sensor evaluation model without screening indicators. First, because there are many evaluation index items, it is not conducive to the evaluator to evaluate and score carefully and accurately; secondly, because the number of independent variables input to the mathematical model is large, and it is difficult to ensure the independence of the independent variables, which leads to the low evaluation accuracy of the model, the maximum relative error of prediction reaches 8.33% as shown in Figure 3(a).
② Single-hidden layer wireless sensor evaluation model for screening indicators. Due to the comprehensive use of the AFP and the questionnaire survey method, the indicators that have an important impact on the evaluation results are screened out, and these evaluation indicators are used as the input of the wireless sensor technology network, which improves the noncorrelation and accuracy of the input independent variables of the network. Therefore, its evaluation accuracy is greatly improved compared with the wireless sensor evaluation model without screening indicators, and the maximum relative error of prediction is 5.12% as shown in Figure 3(b).
③ Double-hidden layer wireless sensor evaluation model for screening indicators. Compared with the single hidden layer, the multi-hidden layer wireless sensor technology network has strong generalization ability and high prediction accuracy [17, 18]. Therefore, this paper also constructs the 8-10-8–1 dual-hidden-layer wireless sensor evaluation model, and the maximum relative error of prediction is 4.13%. Compared with the single-hidden-layer wireless sensor evaluation model, the accuracy is slightly improved as shown in Figure 3(c).
④ GABP evaluation model of screening indicators. Because the principle of genetic algorithm is used to obtain the best initial weight and threshold of wireless sensor neural network, and the important index of screening is used as the input of wireless sensor technology network [19, 20]. The advantages of the algorithm greatly improve the prediction accuracy of the wireless sensor technology network evaluation model, and the maximum relative error of prediction is only 2.49% as shown in Figure 3(d).

## 5. Conclusion

This paper proposes an AHP-based physical education quality evaluation system to address the shortcomings of poor learning generalization ability and large prediction error in wireless sensor technology network-based physical education quality evaluation, in collaboration with domestic scholars to screen important evaluation indicators and optimize wireless sensor technology network algorithm two research directions. The enhanced wireless sensor technology network model based on the genetic algorithm is investigated using the technique's evaluation index system and the questionnaire survey method. The simulation test findings suggest that the teaching evaluation model significantly increases assessment accuracy and predictability and that it has a promising future in teaching management. The assessment accuracy, however, has to be increased because to the tiny amount of network training samples.

## Figures and Tables

**Figure 1:** The steps of improving GA-enabled wireless sensor neural network.

**Figure 2:** Comparison of the prediction error curves of the two networks.

**Figure 3:** (a) Error prediction without screening indicators, (b) error prediction of uni-hidden layer of screening indicators, (c) error prediction of dual-hidden layer of screening indicators, and (d) GABP prediction error for screening indicators.

**Table 1:** Assignment standard of golden scale method.

Scaling	Meaning
1	Two factors *B*_*i*_ and *B*_*j*_ are likewise significant
1.618	Factor *B*_*i*_ is extra significant than *B*_*j*_
2.618	Factor *B*_*i*_ is considerably more significant than *B*_*j*_
4.238	Factor *B*_*i*_ is strongly more significant than *B*_*j*_
Reciprocal of scale	The ratio of the importance of *B*_*i*_ to *B*_*j*_ is the inverse of the ratio of the importance of *B*_*j*_ to *B*_*i*_

**Table 2:** Eight important evaluation indicators based on AHP and questionnaires.

First-level indicator	Serial number	Secondary indicators
Teaching and educating people	X1	Dedication to work, strong sense of responsibility in all aspects of teaching
Teaching organization	X2	The language is standardized, clear, and vivid, and the speed of speech is moderate
Teaching effect	X3	Students can master the basic concepts and principles of the course
	X4	Students enhance analytical problem-solving skills
Teaching content	X5	Highlight important and difficult points, detail properly, and do not follow the script
	X6	Link theory with practice, without discussing content unrelated to the course
Teaching method	X7	Good at interaction, stimulate students' thinking and learning interest
	X8	The teaching ideas are clear and easy to understand, and the methods and means are flexible

## Data Availability

The datasets used and analysed during the current study are available from the corresponding author upon reasonable request.
